# The efficacy of ultrasound treatment as a reversible male contraceptive in the rhesus monkey

**DOI:** 10.1186/1477-7827-10-81

**Published:** 2012-09-12

**Authors:** Catherine A VandeVoort, Theodore L Tollner

**Affiliations:** 1 California National Primate Research Center, University of California, Davis, CA, 95616, USA; 2 Department of Obstetrics and Gynecology, University of California, Davis, CA, 95616, USA; 3 Center for Health and the Environment, University of California, Davis, CA, 95616, USA

**Keywords:** Sperm morphology, Motility, Contraception, Testes, Male reproduction

## Abstract

**Background:**

The use of therapeutic ultrasound as a contraceptive approach has involved nonhuman primates as well as rats and dogs. The current study was undertaken to determine whether this treatment could be a method for reversible contraception, using a model with testes size similar to adult humans.

**Methods:**

Two methods of ultrasound exposure were used, either the transducer probe at the bottom of a cup filled with saline (Cup) or direct application to the surface of the scrotum (Direct). Four adult rhesus (Macaca mulatta) males with normal semen parameters were treated with therapeutic ultrasound at 2.5 W/cm(2) for 30 min. Treatment was given 3 times, one every other day on a Monday-Wednesday-Friday schedule. For each male, semen quality was evaluated a minimum of three times over several months prior to ultrasound exposure and weekly for two months following ultrasound treatment.

**Results:**

Semen samples from all males, regardless of exposure method, exhibited a decrease in the percentage of motile sperm following ultrasound treatment. There was an average reduction in motility of 40% the week following treatment. Similarly, curvilinear velocity and the percentage of sperm with a normally shaped flagellum were also reduced in all males following ultrasound treatment. A significant reduction in the total number of sperm in an ejaculate (total sperm count) was only observed in males that received ultrasound via the cup method. Following treatment via the cup method, males exhibited up to a 91.7% decrease in average total sperm count (n = 2). Sperm count did not approach pre-treatment levels until 8 weeks following ultrasound exposure.

**Conclusions:**

The sustained reduction in sperm count, percent motility, normal morphology, and sperm vigor with the cup exposure method provides proof of principle that testicular treatment with ultrasound can be an effective contraceptive approach in humans.

## Background

Because of the personal, productivity, and societal toll taken by surgery, surgical complications, and the cost of anesthesia, a great need continues to exist for nonsurgical methods of fertility control that are satisfactory, affordable, and consistently available to users. In particular, new methods for men are needed, because currently the only options for men are condoms (which have a high misuse rate and are subject to supply disruptions in low-income countries) and vasectomy (which is surgical and generally permanent). Both surgery and a permanent ending of fertility are psychological barriers for many men. We therefore seek to develop non-permanent, non-surgical methods of contraception for males. Non-surgical, non-invasive methods would also allow efficient and cost-effective use in feral and street populations of animals such as dogs, cats, and monkeys.

The research of Dr. Fahim and colleagues showed brief applications of testicular ultrasound waves to be effective at reducing or eliminating sperm in rats, cats, dogs, rabbits, monkeys, and man [1-6]. Fahim demonstrated that testicular exposure to "low intensity" therapeutic ultrasound, consistent with ultrasound properties applied in physiotherapy of soft tissue and tendon damage [7], for review], resulted in complete and prolonged cessation of sperm production without affecting circulating levels of testosterone [1,2]. In rats, dramatic degeneration of seminiferous tubule epithelium coincided with loss of sperm production and appeared to occur through both temperature-dependent and independent mechanisms following a single 10 min exposure to ultrasound [1]. With dogs and cats, similar effects on tubule morphology and spermatogenesis were observed following two to three serial exposures of ultrasound [2]. Recovery of sperm production to pretreatment levels was observed in both rats and monkeys, depending upon the ultrasound intensity, duration, and coupling medium used in these studies [3,4].

In order to translate this technique to application in men, it is essential to replicate Dr. Fahim’s work to determine first, whether the effect could be confirmed in an independent laboratory with currently available sonicating equipment, and second, if ultrasound could be shown to be an effective method of contraception in a non-human primate species with testes of similar size to those of men. The average testicular volumes of rhesus monkeys (*Macaca mulatta*) chosen for this study were consistent with volumes reported for rhesus monkeys in prior studies [8,9], and within the upper range of testicular volumes measured for healthy adult human males [10,11]. Furthermore, rates of sperm production (based on total sperm numbers in an ejaculate) in rhesus monkeys [12] are similar to average rates of sperm production in proven-fertile men [13]. Therefore, the ability of testicular ultrasound to suppress spermatogenesis in the rhesus monkey is a particularly relevant proof of principle for application of this method in human contraception.

## Methods

### Animals

Four adult male rhesus monkeys (*Macaca mulatta*) were housed at the California National Primate Research Center as pairs in outdoor “corn crib” enclosures. Males were fed Purina monkey chow and water *ad libitum*. Males were sexually mature, ranging in age from 6 to 15 years and in weight from 10 to 15 kg. All procedures for maintenance and handling of the animals were reviewed and approved in advance by the Institutional Animal Use and Care Administrative Advisory Committee at the University of California at Davis. The males were trained to chair restraint, and semen was collected by direct penile stimulation with a Grass 6 stimulator equipped with electrocardiogram pad electrodes (30–50 V, 20 ms duration, 18 pulses/sec) as previously described [12]. Samples were allowed to liquefy for 30 minutes before processing.

Testes volume was determined for all males on the same day, prior to ultrasound exposure. The height (*h*), length (*l*), and width (*w*) of each testis was measured with calipers. The formula for estimating volume of an ellipsoid ( 4/3π x *l*/2 x *w*/2 x *h*/2) was applied to these measurements and averaged across both testes for each male (Table 1).

**Table 1:** Testicular volume (ml) was determined for each male prior to the beginning of the study

**Method**	**Animal**	**Avg. Testicle Vol (ml)**	**% Inhibition of Total Sperm Count**
**Cup**	1	25.1	94.1%
	2	32.1	76.9%
**Direct**	3	35.7	No Inhibition
	4	17.8	49.7%

The % inhibition of total sperm count with treatment was determined for each male by dividing the average total sperm count derived from the first three evaluations following US treatment by the average total sperm count derived from the three pre-treatment semen evaluations x 100.

### Ultrasound exposure

Therapeutic ultrasound treatments were performed with a PHYSIOMED Elecktromedizin AG unit, model: vetri-son portable (Schnaittach, Germany). Exposures were 2.5 W/cm^2^ for 30 min for all males, 3 times, every other day on a Monday, Wednesday, Friday schedule. Two methods of exposure were used: 1) Cup method (N = 2): Animal’s scrotum/testes positioned in the cup and sound waves emitted from the transducer at the base of the cup through a media solution of 3% NaCl before radiating the testes; 2) Direct method (N = 2): Application of the probe directly to the scrotum/testes surface in a continuous, circular manner.

### Semen collection and analyses

Semen samples were collected at weekly intervals from each rhesus monkey; three samples prior to and 9 samples following therapeutic ultrasound exposure. All semen specimens were evaluated according to previously published techniques. Semen volume, sperm density, and percentage of motile sperm were measured according to WHO 1987 methods [14,15]. From these measures, the total sperm count (sperm density x semen volume) and total normal count (sperm density x% morphologically normal sperm) were determined. Ten μl drops of washed sperm were layered onto glass slides, dried, and stained with the method of Papanicolaou [16] and two hundred sperm per specimen were scored for various categories of abnormal forms according to Tollner et al. [17]. For computer assisted measurements of sperm motion characteristics (CASA), sperm were washed and videomicrography was performed as described previously [17,18]. Motion characteristics of the recorded sperm were analyzed with the HTM Ceros, version 10.9d (Hamilton Thorne Biosciences Inc.). At least 200 sperm per semen sample were analyzed for curvilinear velocity (VCL), straight-line velocity (VSL), linearity (LIN), and amplitude of lateral head displacement (ALH).

## Results

Table 1 details the average testicle volume for each male and the percent inhibition of the total sperm count for each male after ultrasound treatment. There were no differences in testicular volume between treatment methods, but the cup methods produced greater inhibition of total sperm count.

The cup method was generally more effective than the direct method (Figures 1 and 2) and suppressed total normal sperm count for 7–8 weeks with a maximal average inhibition of sperm numbers of 93%. The cup method also resulted in a transient reduction of sperm motility and reduced both VCL and ALH, measures of sperm vigor. However, as shown in Figure 2, both methods effectively decreased the total normal sperm count for at least 7 weeks.

**Figure 1:** **Sperm count, sperm morphology, and various sperm motility parameters (percent motility, curvilinear velocity [VCL], and amplitude of lateral head displacement [ALH]) from males treated by either the cup or direct method of ultrasound exposure.** The black arrows indicate the time of ultrasound exposure.

**Figure 2:** **The total number of morphologically normal sperm in an ejaculate (total normal count) from males treated by either the cup or direct method of ultrasound exposure.** The black arrow indicates the time of ultrasound exposure.

Both methods of ultrasound exposure decreased the number of sperm with normal morphology (Figure 1) as well as reduced sample-to-sample variability in the total number of normally shaped sperm (Figure 2). The direct method appeared to have a more pronounced effect on sperm morphology (Figure 1) by increasing the number of sperm with tail defects (Figure 3). As shown in Figures 1 and 2, semen quality recovered within weeks to months following ultrasound treatment. No detectable side effects, such as testicular swelling or redness, or behavior changes were noted with either ultrasound treatment method.

**Figure 3:** Morphology of sperm from males before or after the direct method of ultrasound treatment.

## Discussion

The cup method, a modification of methods used successfully in the rat, the dog, and a smaller primate to suppress spermatogenesis [1,2], results in reduction of semen quality in adult rhesus monkeys. Unlike in other animal models, treatment did not induce azoospermia, yet the numbers of sperm that were vigorously motile and with normal morphology were exceedingly low. Within exposure method, ultrasound treatment appeared to be most effective for males with smaller testes, suggesting that higher levels of exposure may be required to achieve contraception in individuals and animals with greater testicular mass.

Low intensity therapeutic ultrasound has been demonstrated to exhibit both thermal and non-thermal effects on tissue. It has been well established that acoustic absorption by tissue can result in elevated tissue temperature; the rate at which temperature rises is proportional to the intensity of the ultrasonic beam and inversely proportionate to the density and heat capacity of the tissue [7]. Effects believed to arise from low intensity (0.125–3 W/cm^2^) ultrasound-induced heating include changes in blood flow, increased flexibility of tendons and scar tissue, and decrease in joint stiffness [7]. Independent of temperature, acoustic radiation produces a time-averaged force that can act on objects in an acoustic field [19], for review]. Acoustic radiation forces can induce the rotation or spinning of particles as well as produce flow or streaming of fluids. Streaming can alter the local environment of a cell, resulting in altered concentration gradients across cellular membranes [7]. Radiation forces underlie a number of bioeffects including stimulation of cardiac and neural tissue, acceleration of bone healing, enhancement in collagen synthesis, and improvement in both drug uptake by cells (sonoporation), and transdermal delivery of drugs (sonophoresis) [19].

It is not entirely clear how ultrasound affects sperm production. Increased testicular heat alone has been shown to slow spermatogenesis, induce apoptosis in developing sperm cells, and lead to lower numbers of motile and morphologically normal spermatozoa in an ejaculate [20], for review]. From rodent and livestock studies, the cells that are most susceptible to damage by acute heat stress are pachytene spermatocytes and spermatids, although B spermatogonia can also be damaged if degree and duration of heat exposure are increased [21], for review]. In men, elevated scrotal temperatures due to lifestyle, workplace environment, varicocele, or cryptorchidism are inversely correlated with sperm quality [22-24]. From Fahim's work and Tsuruta's studies in the rat, brief exposures of the testes to low intensity ultrasound result in an increase in intratesticular and scrotal temperatures ranging from one up to several degrees Celsius above body temperature [1,2,6,25]. Similarly elevated temperatures can be achieved by warming testicles in a water bath for 15 to 30 minutes, but the effect on sperm production is not nearly as pronounced as when ultrasound is applied [1,25]. The mechanisms of the extra-temperature effects observed in testicular tissue with ultrasound treatment, however, are not fully understood. Fahim demonstrated that ultrasound exposure results in changes in electrolyte concentrations in fluid from seminiferous tubules and rete testes [3]. Perhaps this finding speaks to ultrasound-induced alterations in the transport of substances across the tubule that may contribute to the stress of spermatogenic cells.

In our study, we demonstrate that the cup method, using warm saline as a coupling medium, is more effective at suppressing sperm production than direct application of the ultrasound probe to the scrotum. Initially, we found this to be a surprising result as we expected the cup method to produce more ultrasound beam scattering and therefore less focused propagation of ultrasound energy through testicular tissue. Moreover, similar conditions of direct application, reproduced by the same model of sonicator, were applied to the testes of dogs and resulted in azoospermia in all animals treated [26]. This discrepancy in response, as well as the lack of a consistent effect with either cup or direct methods, might be explained by differences in testes size between and within species and a general tendency of the testes to resist temperature change due to gonadal vascular and scrotal muscular and glandular mechanisms [20].

Differences in testes size may account, at least in part, for the differences in efficacy that we see with ultrasound in the rhesus monkey. In both treatment methods, the male with the smaller testes exhibited the greatest reduction in sperm numbers following ultrasound. We speculate that the methods we tested did not sufficiently elevate intratesticular temperatures in males with greater testicular mass. Potentially for this reason, the cup method was superior to the direct because it provided conditions (saline bath maintained at 35-37°C) whereby testicular temperature should stay elevated during the duration of ultrasound exposure. Evidence for this possibility is provided in the rat, where the temperature of the conducting medium was an important factor for observing maximal effects with ultrasound [25]. When saline in the ultrasound treatment cup was maintained at 37°C, the intratesticular temperature in the rat rose rapidly (within 1–2 minutes of ultrasound exposure) above body temperature [25]. By contrast, the direct method in the monkey, by not controlling ambient temperature, likely could not overcome scrotal mechanisms for liberating heat from the testes. It should also be noted that the testes of the monkeys used in our study on average were three times larger (by volume) than testes of the dogs used by Leoci et al. [26], and adult rhesus monkey testes in general are approximately 15 times larger (by mass) than testes of sexually mature rats [27-29]. It is therefore not surprising that similar ultrasound protocols might not produce highly similar results among species that vary widely with respect to testicle size.

An important finding of the present study is that the effects of ultrasound appear to be fully reversible. The sperm quality of all males, independent of treatment method, recovered somewhat sharply to pretreatment levels between week seven and week nine following ultrasound exposure. This trend was particularly dramatic for male #1, where sperm production was nearly eliminated (total sperm count and normal sperm count were inhibited by over 99%) in the initial weeks post treatment. Fahim reported a similarly robust recovery in sperm production following testicular ultrasound with the smaller cynomolgus monkey (*Macaca fascicularis*) [3]. Together these studies suggest that primate testes may be particularly resilient to ultrasound radiation, with full recovery of spermatogenic potential. If equally true for men, ultrasound could prove viable as a non-invasive reversible contraceptive provided the duration of prophylaxis can be extended. Additional studies in non-human primates are needed to determine optimal exposure conditions, perhaps including an increase in the ambient temperature, to ensure a prolonged knockdown of spermatogenesis to levels that would be consistent with providing effective contraception.

A concern with any treatment that results in heat stress of the testes is the potential of DNA damage in sperm. Mild, acute, scrotal heat stress leads to DNA strand breaks in spermatogenic cells in mice [30,31]. Many of these sperm progenitors are eliminated by apoptosis, but as many as 70% of the sperm that developed from thermal-damaged spermatocytes have chromatin abnormalities indicative of DNA defects [32]. In vivo and in vitro fertilization with these sperm results in numerous embryonic abnormities and sharply reduced rates of blastocyst formation [32]. These studies mirror a growing concern in the field of reproductive medicine that certain long-term health adversities seen in children are potentially associated with conception achieved with sperm possessing damaged DNA [33]. Before ultrasound treatment should be considered as a method of reversible contraception in humans, future studies should determine whether DNA damage persists in spermatozoa following recovery of sperm numbers and normal morphology in the months following testicular ultrasound exposure.

## Conclusions

We confirm in a non-human primate species with testicles that compare in size with those of men that ultrasound treatment results in reduced sperm numbers and quality. This study provides a proof of principle that testicular ultrasound exposure has the potential to be a viable approach for contraception in humans.

## Competing interests

The authors declare that they have no competing interests.

## Authors’ contributions

CV and TT were involved in all aspects of this study, including design, treatment and coordination as well as various semen analyses and preparation of the manuscript. Both authors read and approved the final manuscript.
